# National Lupus Hospitalization Trends Reveal Rising Rates of Herpes Zoster and Declines in Pneumocystis Pneumonia

**DOI:** 10.1371/journal.pone.0144918

**Published:** 2016-01-05

**Authors:** Sara G. Murray, Gabriela Schmajuk, Laura Trupin, Lianne Gensler, Patricia P. Katz, Edward H. Yelin, Stuart A. Gansky, Jinoos Yazdany

**Affiliations:** 1 Department of Medicine, University of California San Francisco, San Francisco, California, United States of America; 2 Department of Medicine, Veterans Administration, San Francisco, California, United States of America; 3 Phillip R. Lee Institute for Health Policy Studies, University of California San Francisco, San Francisco, California, United States of America; 4 Division of Oral Epidemiology and Dental Public Health, Department of Preventive and Restorative Dental Sciences, University of California San Francisco, San Francisco, California, United States of America; Instituto de Higiene e Medicina Tropical, PORTUGAL

## Abstract

**Objective:**

Infection is a leading cause of morbidity and mortality in systemic lupus erythematosus (SLE). Therapeutic practices have evolved over the past 15 years, but effects on infectious complications of SLE are unknown. We evaluated trends in hospitalizations for severe and opportunistic infections in a population-based SLE study.

**Methods:**

Data derive from the 2000 to 2011 United States National Inpatient Sample, including individuals who met a validated administrative definition of SLE. Primary outcomes were diagnoses of bacteremia, pneumonia, opportunistic fungal infection, herpes zoster, cytomegalovirus, or pneumocystis pneumonia (PCP). We used Poisson regression to determine whether infection rates were changing in SLE hospitalizations and used predictive marginals to generate annual adjusted rates of specific infections.

**Results:**

We identified 361,337 SLE hospitalizations from 2000 to 2011 meeting study inclusion criteria. Compared to non-SLE hospitalizations, SLE patients were younger (51 vs. 62 years), predominantly female (89% vs. 54%), and more likely to be racial/ethnic minorities. SLE diagnosis was significantly associated with all measured severe and opportunistic infections. From 2000 to 2011, adjusted SLE hospitalization rates for herpes zoster increased more than non-SLE rates: 54 to 79 per 10,000 SLE hospitalizations compared with 24 to 29 per 10,000 non-SLE hospitalizations. Conversely, SLE hospitalizations for PCP disproportionately decreased: 5.1 to 2.5 per 10,000 SLE hospitalizations compared with 0.9 to 1.3 per 10,000 non-SLE hospitalizations.

**Conclusions:**

Among patients with SLE, herpes zoster hospitalizations are rising while PCP hospitalizations are declining. These trends likely reflect evolving SLE treatment strategies. Further research is needed to identify patients at greatest risk for infectious complications.

## Introduction

Infection is one of the leading causes of morbidity and mortality in patients with systemic lupus erythematosus (SLE), and it is estimated that 14–52% of SLE hospitalizations are for infection [1–3]. In a review of consecutive SLE patients seen in the ambulatory setting, approximately 15% of patients had previous infections that were serious enough to result in hospitalization and 25% of all deaths in this cohort were due to infection [4]. While pneumonia has been shown to be the leading cause of preventable hospitalization in patients with SLE, opportunistic infections such as pneumocystis pneumonia (PCP) are associated with mortality as high as 46% [5,6]. Debilitating viral infections, such as herpes zoster and cytomegalovirus (CMV), are also seen at significantly higher rates in patients with SLE [7–12].

Immunosuppressive practices in SLE have evolved over the past fifteen years. For example, in the case of lupus nephritis, a common and life-threatening manifestation of SLE, therapies have evolved to include increasing use of mycophenolate mofetil (MMF) and lower cumulative dose cyclophosphamide [13–15]. Although it is plausible that evolving immunosuppressive regimens would change the profile of infectious complications in SLE, it is unclear how trends in hospitalizations for infections have changed over the same time period.

To address this question, we evaluated trends in infections associated with SLE hospitalizations between 2000 and 2011 in the National Inpatient Sample. Specifically, we evaluated the prevalence of serious and opportunistic infections in patients with SLE, including bacteremia, pneumonia, opportunistic fungal infections, herpes zoster, CMV, and PCP. In the general medical literature, reported rates of hospitalizations for severe infections such as sepsis are rising for unclear reasons [16–18]. We therefore evaluated trends in infectious complications of SLE over time in comparison with the general non-SLE hospitalized population, with the aim of identifying whether there might be trends that are unique to SLE.

## Materials and Methods

### Study population

Data were derived from the United States (US) Healthcare Cost and Utilization Project National Inpatient Sample (NIS), a de-identified database that includes 20% of all hospital discharges in the United States. The NIS contains data on demographics, resource-utilization, and some clinical parameters, including one primary and up to 24 secondary International Classification of Disease-9 Clinical Modification (ICD-9) discharge diagnoses.

We analyzed all available hospital discharges between 2000 and 2011 with an ICD-9 code for SLE (710.0) as the primary or secondary diagnosis, a validated administrative definition[19]. The control group comprised a 1% random sample of non-SLE hospitalizations from each year over the same time period. All included discharges were for individuals who were 18 years of age or older. We excluded hospitalizations from both the SLE cohort and the non-SLE control cohort if they carried an ICD-9 code related to pregnancy or human immunodeficiency virus (HIV). We also excluded hospitalizations that were missing covariates of interest; the only covariate with more than 1% missing data was race/ethnicity, discussed below.

### Outcomes and covariates

We evaluated the prevalence of several clinically relevant infections among patients with SLE as our primary outcomes. These included a diagnosis of bacteremia, pneumonia, opportunistic fungal infections, herpes zoster, CMV, and PCP. Prevalent bacteremia (038.x, 790.7) and pneumonia (481.x, 482.x, 483.x, 484.x, 485.x, 486.x., 513.0, 003.22) were identified by previously validated ICD-9 codes[20,21]. Opportunistic fungal infections were defined using ICD-9 codes for candidiasis (112.5, 112.81, 112.83, 112.84), coccidiomycosis (114.x), Cryptococcus (117.5, 321.0), aspergillus (117.3, 484.6), and histoplasmosis (115.x), and excluding codes for allergic bronchopulmonary aspergillosis and candidiasis of the lung to maximize the specificity of this definition as previously described[22,23]. Herpes zoster was identified by ICD-9 code 053.x and CMV was identified by ICD-9 code 054.x[24]. Finally, PCP was identified by ICD-9 code 136.3 as previously described[6,25].

Covariates included age, gender, race/ethnicity (White, Black, Hispanic, other, and missing) and a modified Charlson comorbidity score[26,27]. The modified Charlson score was computed for each hospitalization as previously described, excluding rheumatic disease[26,27].

To address the fact that 15–20% of states do not report race/ethnicity, we conducted three sensitivity analyses: (1) assuming all missing hospitalizations were White, (2) assuming all were Black, and (3) excluding these hospitalizations entirely, which is tantamount to assuming the racial/ethnic proportions were the same as in the non-missing data. Trends remained the same regardless of the approach to handling missing data (data not shown).

### Statistical Analyses

We performed cross-sectional Poisson regression (including years 2000–2011) to establish prevalence ratios for specific infectious complications in SLE hospitalizations compared with non-SLE hospitalizations. We chose Poisson regression because outcomes were rare. Separate regression analyses were performed for each infectious outcome of interest, and each was adjusted for the covariates listed above.

To evaluate trends over time among SLE hospitalizations, we used Poisson regression including year (2000–2011) as an independent variable. To evaluate trends over time in SLE hospitalizations compared with non-SLE hospitalizations, we used Poisson regression with an effect modification term for SLE and year (i.e. interaction of SLE and year). These regression analyses were adjusted for covariates. We used predictive marginals, a model-based approach for generating standardized estimates, to calculate annual adjusted rates for each infectious outcome in both the SLE and non-SLE hospitalized populations. We graphically represented those estimates for each year between 2000 and 2011. In order to understand whether the change in prevalence over time was disproportionate in SLE hospitalizations, we calculated adjusted prevalence ratios for each infectious outcome by dividing the adjusted rates in the SLE cases by the adjusted rate in non-SLE hospitalized populations for each year, and graphed the prevalence ratios from 2000 to 2011. Linear contrasts were used to calculate difference in differences with confidence intervals for the change in infection rate over time in SLE hospitalizations compared with non-SLE hospitalizations.

## Results

We identified 375,125 hospitalizations for adult patients (≥18 years old) with SLE, between 2000 and 2011 in the NIS. From this cohort, we excluded those with a diagnosis code for pregnancy (n = 12,811) and those with HIV (n = 907). We also excluded hospitalizations when the data set did not include gender (n = 74). Because some states in the NIS do not report race/ethnicity, 69,378 (19%) of SLE hospitalizations were missing this covariate and were coded as such as described above. Ultimately, 361,337 hospitalizations with SLE were included in our analyses. The 1% randomly selected control group included 668,267 non-SLE hospitalizations. Details on the underlying cohort from which the control group was selected (excluding pregnancy-related conditions and HIV) can be found in the HCUP Statistical Briefs [28].

Characteristics of SLE and non-SLE hospitalizations between 2000 and 2011 are shown in Table 1. Hospitalizations for SLE had a mean age of 51 and 89% were female, compared to hospitalizations without SLE that had a mean age of 62 and 54% were female. The mean modified Charlson score was similar in hospitalizations with and without SLE, 1.6 and 1.4 respectively. Amongst SLE hospitalizations in which race/ethnicity was identified, 44% were White, 23% were Black and 9% were Hispanic. In contrast, 57% of persons without SLE who were hospitalized were White, while only 11% were Black and 7% were Hispanic.

**Table 1:** Characteristics of SLE and non-SLE hospitalizations in the National Inpatient Sample, between years 2000 and 2011.

	Non-SLE*	SLE
	(N = 668,267)	(N = 361,337)
**Age, years**	62 ± 19	51 ± 17
**Female, %**	54%	89%
**Charlson comorbidity score, mean**	1.4 ± 1.6	1.6 ± 1.9
**Race/ethnicity, %**		
** White**	57%	44%
** Black**	11%	23%
** Hispanic**	7%	9%
** Other**	4%	4%
** Missing**	22%	19%

SLE = systemic lupus erythematous.

*Represents a random 1% sample of all non-SLE NIS hospitalizations between 2000 and 2011.

The prevalence of specific infections amongst hospitalizations with and without SLE are shown in Table 2. Pneumonia was the most prevalent infectious complication measured, present in 9.5% of SLE hospitalizations and 8.0% of non-SLE hospitalizations. PCP was the most rare, occurring in 0.04% of SLE hospitalizations compared with 0.01% of non-SLE hospitalizations. In adjusted Poisson regression analyses, all specific infections were significantly more prevalent among SLE hospitalizations compared to non-SLE hospitalizations (see Table 2). As indicated by prevalence ratios (PR), the greatest differences between persons with and without SLE who were hospitalized were observed for opportunistic fungal infections (PR 2.7, 95% CI 2.6 to 2.9), herpes zoster (PR 2.5, 95% CI 2.4 to 2.7), CMV (PR 3.7, 95% CI 3.1 to 4.5), and PCP (PR 3.3, 95% CI 2.4 to 4.6).

**Table 2:** Prevalence of specific infections in SLE hospitalizations compared with non-SLE hospitalizations in the National Inpatient Sample, between years 2000 and 2011.

	Prevalence of infection among hospitalizations		Adjusted prevalence ratio (95% CI) in SLE hospitalizations**
	Non-SLE*, N (%)	SLE, N (%)	
**Bacteremia**	28,606 (4.3%)	23,008 (6.4%)	1.7 (1.6–1.7)
**Pneumonia**	53,366 (8.0%)	34,398 (9.5%)	1.5 (1.5–1.6)
**Opportunistic Fungal**	1,746 (0.3%)	2,658 (0.7%)	2.7 (2.6–2.9)
**Herpes Zoster**	1,825 (0.3%)	2,247 (0.6%)	2.5 (2.4–2.7)
**Cytomegalovirus**	169 (0.03%)	482 (0.13%)	3.7 (3.1–4.5)
**Pneumocystis Pneumonia**	69 (0.01%)	129 (0.04%)	3.3 (2.4–4.6)

SLE = systemic lupus erythematous.

*Represents a random 1% sample of all non-SLE NIS hospitalizations between 2000 and 2011.

**Prevalence ratios for specific infections are derived from individual Poisson regression analyses, adjusted for age, gender, race/ethnicity, and a modified Charlson score.

We then evaluated whether the prevalence of infections among SLE hospitalizations changed over time. In both unadjusted and adjusted Poisson regression analyses, the prevalence of each specific infection varied with the year. In adjusted analyses of SLE hospitalizations, rates of infection were increasing by approximately 3% per year for bacteremia (95% CI 2% to 3%), 1% per year for pneumonia (95% CI 1% to 2%), 1% per year for opportunistic fungal infections (95% CI >0% to 2%), 4% per year for herpes zoster (95% CI 2% to 5%), and 5% per year for CMV (95% CI 2% to 8%). On the contrary, the rate of PCP was decreasing by approximately 7% per year (95% CI -2% to -13%).

Because reported rates of sepsis and severe infections are rising in the general hospitalized population [16–18], we sought to identify whether the change in prevalence of specific infections over time in SLE-related hospitalizations was different than that seen in non-SLE hospitalizations. Annual adjusted rates of specific infections for SLE and non-SLE related hospitalizations between 2000 and 2011 are shown in Fig 1. Although the rate of many infectious complications, including bacteremia, pneumonia, opportunistic fungal infections, herpes zoster, and CMV increased over the eleven year period in SLE related hospitalizations, the increase was disproportionate to non-SLE related hospitalizations only for herpes zoster. Based on adjusted regression analyses with an interaction term for a diagnosis of SLE and year, between 2000 and 2011, rates of herpes zoster increased by 44% in SLE hospitalizations and only 17% in non-SLE hospitalization, with a significant and positive difference in differences of 22% (95% CI >0% to 49%). Other infections showed a negative or insignificant difference in differences. For PCP, where rates of infection were clearly declining in SLE-related hospitalizations, the interaction of SLE and year was also significant in the entire cohort: between 2000 and 2011 there was an 227% decrease in PCP in SLE-related hospitalizations while there was a 29% increase in non-SLE hospitalizations, with a significantly negative difference in differences of 292% (95% CI 115% to 744%). Fig 2 summarizes PRs for select infections, including pneumonia, herpes zoster, CMV, and PCP. The PRs for herpes zoster increased in SLE related hospitalizations while they declined for PCP.

**Fig 1:** Annual adjusted rates of specific infections per 10,000 hospitalizations, among hospitalizations with SLE compared with non-SLE hospitalizations, between 2000 and 2011 in the NIS. Annual rates of infections are adjusted for age, gender, race/ethnicity, and a modified Charlson score.

**Fig 2:** Adjusted annual prevalence ratios for specific infections in SLE hospitalizations compared with non-SLE hospitalizations in the NIS.

## Discussion

In this large, national United States study of hospitalizations for infectious complications of SLE, we found that a diagnosis of SLE was associated with increased measured severe and opportunistic infections, including bacteremia, pneumonia, opportunistic fungal infections, herpes zoster, CMV, and PCP. We also found that among SLE hospitalizations, rates of all these infections significantly rose between 2000 and 2011, with the exception of PCP which significantly declined. Notably, herpes zoster was the only infection that disproportionately increased over time among SLE-hospitalizations when compared with non-SLE hospitalizations.

A higher incidence of herpes zoster has been reported in SLE in several studies. Both the use of immunosuppression and immune dysregulation that is a consequence of the disease are thought to contribute [7,9,29,30]. While cellular immune response to the virus may be impaired regardless of immunosuppressive regimen, multiple studies have demonstrated that medications used to treat SLE, including prednisone, azathioprine, mycophenolate mofetil, and cyclophosphamide, increase the risk of herpes zoster infection [7,9,12,29,30]. In a recent large prospective cohort study of 1485 patients with SLE, the hazard ratio for an incident diagnosis of herpes zoster was greatest (hazard ratio 5.00, 95% CI 1.40–17.60) in SLE patients taking mycophenolate mofetil, followed by prednisone [7]. Use of mycophenolate mofetil for induction and maintenance of lupus nephritis and for severe non-renal lupus has become increasingly widespread over the past fifteen years, with multiple clinical trials and a meta-analysis demonstrating equivalence to cyclophosphamide for induction therapy [14,15,31,32]. We hypothesize that the increasing rate of hospitalization with herpes zoster seen in our study reflects this evolution of clinical practice.

It is interesting that the rate of PCP is declining among SLE hospitalizations. PCP is a rare but greatly feared complication of immunosuppression, as it presents more aggressively in patients with connective tissue disease when compared with HIV patients and has a mortality rate of approximately 40–45% [6,33]. Previous studies indicate that a dose of glucocorticoids ≥16mg increases the risk of PCP in non-HIV individuals [34]. A review of the literature involving 76,156 SLE patients on cyclophosphamide reported a PCP prevalence of 0.16% [35]. In this same manuscript, a survey of rheumatologists found that prophylactic practices varied widely, with only 50% of rheumatologists using routine PCP prophylaxis in SLE patients treated with cyclophosphamide [35]. Similar to trends seen in herpes zoster, the declines in PCP seen in our study may also represent declining use of cyclophosphamide and increasing use of mycophenolate. The Euro-Lupus Nephritis Trial demonstrated equivalent efficacy and a favorable side-effect profile for low-dose intravenous cyclophosphamide compared with a previously standard high-dose regimen [13,36]. Recently published American College of Rheumatology guidelines reflect these landmark trials, and recommend mycophenolate or cyclophosphamide for induction of class III/IV lupus nephritis, with lower cumulative-dose “Euro-Lupus” dosing of cyclophosphamide, and mycophenolate or azathioprine for maintenance therapy [37]. While all of these medications are felt to be immunosuppressive, interestingly, both animal studies and data from renal transplant trials suggest that mycophenolate may have antimicrobial properties that protect against PCP, although data specific to lupus patients is lacking [38–40]. Because of the risk of serious adverse events associated with antimicrobial prophylaxis for PCP, it is recommended that prophylaxis only be used when the risk of PCP is greater than 3.5% [41]. Additional studies are needed to determine which SLE patients using modern immunosuppressive regimens are truly at risk and warrant prophylaxis.

This is one of the largest population-based studies evaluating hospitalization trends in specific serious and opportunistic infections in SLE to date. Our approach addresses some of the limitations of previous research regarding infections and lupus, including a recent report by Tektonidou et al. evaluating trends in hospitalizations for general infections in SLE also using the NIS [42]. This study found significantly higher relative risks for hospitalizations for all infections, all of which increase dramatically relative to the non-SLE population. However, a limitation of this approach relates to the use of standardization from a population-based cohort that may not necessarily be representative of the entire U.S. population (given that the population is mostly African-American and Caucasian). Furthermore, the study generated rates by standardization to 2000 US census estimates, which don’t take into account population changes over time or increasing rates of all-cause hospitalizations in both SLE and non-SLE populations. In our study, adjusted rates of infection in SLE and non-SLE hospitalizations were generated in comparison with all hospitalizations. It is for these reasons that we believe our results more accurately represent underlying trends in infection for SLE hospitalizations, reflecting truly disproportionate changes in rates Herpes Zoster and PCP over time.

While the NIS provides us with a large representative sample of the entire hospitalized US population in which we can study rare infectious outcomes, it is not without limitations. Identifying diagnoses through ICD-9 codes may result in misclassification, although non-differential misclassification of outcome generally biases a study towards null findings. Evaluating trends over time raises concern that reported trends may represent changes in coding and billing practices rather than the true rate of disease. This phenomenon has been observed in the general medical literature, where rates of hospitalization for sepsis appear to be rising, but mean cost per case and case-related mortality appears to be declining [16–18]. While these observed trends could represent improved diagnosis and care, it is also possible that they represent changes in reimbursement formulas associated with efforts to enhance coding practices. Thus, we chose to use those hospitalized for reasons other than SLE as a control group, and found herpes zoster and PCP as the two diseases where changes are truly disproportionate in SLE.

Our study captures infections associated with hospitalizations, and may not be representative of less severe infections. It is impossible to know the severity of a given infection, whether infection was the reason for initial presentation or whether it was a complication of the hospitalization. There is also no way to track repeat admissions over time. Additional limitations of the NIS are that it lacks medications and laboratory values, and we cannot track individual patients over time. We therefore could not quantify the degree of immunosuppression or whether patients were receiving antimicrobial prophylaxis. Future studies using data sources such as electronic health record data repositories are warranted to further understand the relationship between SLE, immunosuppressive drug use and infection.

In conclusion, the prevalence of herpes zoster in SLE-related hospitalizations is increasing, while the prevalence of PCP in such hospitalizations has declined significantly. Given the time period of this study, the rise in herpes zoster may be a consequence of the advances in our treatment of lupus nephritis and non-renal lupus. Studies are currently underway to evaluate the safety and efficacy of herpes zoster vaccination in patients with SLE, and the vaccine appears to be safe in patients with mild disease who are taking only mild to moderate immunosuppressive medication [43]. It is also worth considering whether patients at greater risk would benefit from antiviral prophylaxis for both herpes zoster and cytomegalovirus, given the success of this strategy in solid organ and hematopoietic transplants [44]. In contrast, because SLE patients are at very minimal risk of PCP and this risk appears to be declining, it is also worth considering whether our use of antimicrobial prophylaxis for this rare disease should be reexamined, particularly given the increased prevalence of sulfa drug allergy in SLE patients[45]. Future studies that draw upon the richness of clinical information available in the electronic medical record and allow for large multi-center collaborations will provide the data necessary to develop algorithms that truly prognosticate these rare but severe infectious outcomes. In the meanwhile, selecting minimally immunosuppressive drug regimens, vaccinating patients when appropriate, and counseling patients and providers on rigorous infectious control practices will likely mitigate risk.
